The article "A Comprehensive Review on Smart Health Care: Applications, Paradigms, and Challenges with Case Studies" was published in 2022. Journal: Contrast Media Mol Imaging.

# A Comprehensive Review on Smart Health Care: Applications, Paradigms, and Challenges with Case Studies

**DOI:** 10.1155/2022/4822235

**Published:** 2022-09-29

**Authors:** Syed Saba Raoof, M. A. Saleem Durai

**Affiliations:** SCOPE, Vellore Institute of Technology, Katpadi, Vellore 632014, Tamilnadu, India

## Abstract

Growth and advancement of the Deep Learning (DL) and the Internet of Things (IoT) are figuring out their way over the modern contemporary world through integrating various technologies in distinct fields viz, agriculture, manufacturing, energy, transportation, supply chains, cities, healthcare, and so on. Researchers had identified the feasibility of integrating deep learning, cloud, and IoT to enhance the overall automation, where IoT may prolong its application area through utilizing cloud services and the cloud can even prolong its applications through data acquired by IoT devices like sensors and deep learning for disease detection and diagnosis. This study explains a summary of various techniques utilized in smart healthcare, i.e., deep learning, cloud-based-IoT applications in smart healthcare, fog computing in smart healthcare, and challenges and issues faced by smart healthcare and it presents a wider scope as it is not intended for a particular application such aspatient monitoring, disease detection, and diagnosing and the technologies used for developing this smart systems are outlined. Smart health bestows the quality of life. Convenient and comfortable living is made possible by the services provided by smart healthcare systems (SHSs). Since healthcare is a massive area with enormous data and a broad spectrum of diseases associated with different organs, immense research can be done to overcome the drawbacks of traditional healthcare methods. Deep learning with IoT can effectively be applied in the healthcare sector to automate the diagnosing and treatment process even in rural areas remotely. Applications may include disease prevention and diagnosis, fitness and patient monitoring, food monitoring, mobile health, telemedicine, emergency systems, assisted living, self-management of chronic diseases, and so on.

## 1. Introduction

The most indispensable aspect of life is undeniably health. In recent years, advanced healthcare systems have gained immense popularity due to demographic growth, and an increase in diseases which, in turn, requires enormous clinical assets and even hospital staff. Therefore, it challenges tremendous, computerized health systems providing excellent services to both patients and the hospital staff as traditional healthcare systems are incompetent to accomplish the necessity of all humans as it is not affordable and accessible to everyone. Advancement in the medical area was initiated in the early 1991s and it was considered a completely advanced area for treatment. Since then, healthcare systems had been revolutionized in several ways, for example, agile treatment, appropriate early patient serving, delivering, and monitoring healthcare services remotely, and quick action towards emergency cases. The key challenge encountered during the advancement of the medical area was its demand for emerging efficient types of equipment to deliver the best services to patients [1]. This challenge can be addressed by employing IoT and evolutionary technologies. Implementation of IoT in the medical area gained popularity, following modern techniques like smart cities, smart regions, and smart devices.

The article "A Comprehensive Review on Smart Health Care: Applications, Paradigms, and Challenges with Case Studies" was published in 2022. Journal: Contrast Media Mol Imaging.

IoT achieved immense popularity because of its data acquiring and visualizing property through sensing the objects and communication with devices through wireless networks. IoT devices are capable of sensing, visualizing, collecting, and sharing data, and communication among the devices can be done by wireless IoT protocols like Bluetooth, ZigBee, *Z*-Wave, WiFi, and RFID [2, 3]. These protocols play a vital role in the healthcare sector since they ensure ease and flexibility for data communication and data monitoring among employed devices. Data collected from these devices are used for different tasks like disease classification, designing, patient monitoring, and so on. In remote areas where one cannot access the hospital services suffers a lot, and this leads to worsening the patient condition; this situation can be handled by new emerging technology, i.e., tiny wireless chips or sensors connected with IoT devices remotely monitors patient's health [4]. Wired or wireless sensors [5] connected to the patient's body acquire securely patient data and at the same time physicians have access to data; thus, it provides ease for decision making. IoT applications in the healthcare sector benefit everyone to access medical help remotely, enhance the duration of therapy, and affordable cost. Many researchers had implemented various smart health devices like health monitoring and controlling, smart thermometers, automated insulin delivery (AID) systems [6], remote care biometric scanners, sleep monitoring, monitoring drug interaction, and so on.

Regardless of this progress (i.e., IoT in healthcare), there are still challenges to overcome like deploying of IoT system which can manage a large amount of data along with proving all security concerns like data confidentiality, integrity control, authorization, and authentication.

Cloud concepts also play a vital role in smart healthcare systems. It provides firm and efficient access to data; storage can be done effectively, and the above-mentioned challenges can be overcome by employing cloud services [7]. Deep learning (DL) techniques like Convolutional Neural Networks (CNN), Autoencoders (AE), Deep Belief Networks (DBNs), Long Short-Term Memory (LSTM), Recurrent Neural Networks (RNNs), etc. [8, 9] are being employed to analyze large data and to effectively detect and diagnose various diseases. DL applications in medical imaging and medical signals assist both physicians and patients effectively. Integrating IoT technologies along with cloud services, machine learning, and deep learning techniques enhances smart healthcare services immensely [10].

The article "A Comprehensive Review on Smart Health Care: Applications, Paradigms, and Challenges with Case Studies" was published in 2022. Journal: Contrast Media Mol Imaging.

The key objective of this research paper is to provide a comprehensive survey related to IoT-cloud-Artificial Intelligent-Machine Learning-Deep learning healthcare systems (i.e., smart healthcare). The rest of the study is organized as follows: Section 2 discusses related work. Section 3 explains background study. Section 4 discusses smart healthcare applications. Section 5 challenges in smart healthcare systems. Section 6 explains conclusion and Table 1 describes the abbrevations.

## 2. Related Work

This section provides a review of some existing smart healthcare papers and Table 2 demonstrates the summary survey carried out during our research work.

Ali et al. [11] developed a Smart Healthcare Monitoring System (SHMS) to predict heart disease by employing deep ensemble learning, and feature fusion methods. For experimental analysis, both sensor data and EMR data had been utilized and the system obtained 98.5% accuracy in predicting heart disease. The entire process is carried out in four layers, i.e., data collection layer, data fusion and feature extraction layer, data preprocessing layer, and prediction layer. Ismail et al. [12] proposed an efficient solution “a smart speech recognition system” for elderly and disabled patients. The main components of the proposed system are smartphones, controlling devices, and household appliances/devices. A combination of support vector machine (SVM) and dynamic time wrapping (DTW) approaches had been used for speech recognition and controlling the system Raspberry Pi board, which recorded 97% accuracy. Rizwan et al. [13] introduced an integrated smart system (i.e., deep neural network (DNN) + IoT) namely Grey Filter Bayesian Convolutional Neural Network (GFB-CNN) depending on real-time analytics for analyzing heart signals. Cloud services had been also used for data storing and sharing. Mobile HEALTH (MHEALTH) dataset had been utilized and obtained 88% of accuracy. Subasi et al. [14] implemented efficient and automated Human Action Recognition (HAR) system by employing various ML algorithms like SVM, K-NN, ANN, Naive Bayes, RF, CART, C4.5, REP Tree, and LAD Tree, and compared the results of all these algorithms and recorded accuracy between 84% and 99%. Body sensor data REALDISP and Smartphone sensor data are used for experimental analysis of the system. Pereira et al. [15] implemented a 3D-UNet model for brain disease classification and the BRATS dataset is used and achieved 89% accuracy. Further interpretability techniques were employed for analyzing prediction which enhanced preprocessing step.

The article "A Comprehensive Review on Smart Health Care: Applications, Paradigms, and Challenges with Case Studies" was published in 2022. Journal: Contrast Media Mol Imaging.

Manogaran et al. [16] proposed MF-R and GC architecture for monitoring patients' health. The proposed architecture is composed of three phases, i.e., data collection, transfer, and storage phase. The system monitors blood pressure, heart rate, sugar level, respiratory rate, and body temperature. Stochastic gradient descent algorithm and logistic regression techniques are employed in the proposed smart system for detecting heart diseases and the CHDD dataset is used for this purpose. Vikas and Ananthula [17] designed a network, namely Body Sensor Network (BSN) for monitoring the health condition of patients and LabView software is employed on the patient side. The proposed model helps physicians to view and monitor the patient's health remotely. Arduino board is used for connecting the sensors to acquire patient health data. Luca et al. [18] developed IoT-based and Smart Health Care System (SHS) architecture for monitoring patient health, tracking hospitals' biomedical devices, and nursing staff in nursing institutes. CoAP, REST, and 6LoWPAN, IoT paradigms are employed to allow intercommunication and interoperation between SHS devices (i.e., UHF, WSN, and phones). The proposed system is divided into two subsystems: one to monitor patients and the other to deal with emergencies. Loubet et al. [19] developed a Cyber-physical system for structural patient health monitoring. Smart mesh WSN consisting of sensing and communication nodes and a far-field Wireless Power Transmission system (a battery and wire-free system) is used to develop the proposed architecture. Autonomous control of sensing nodes is made possible because of Wireless Power Transmission. Swati et al. [20] proposed a block-wise fine-tuning method using a pretrained CNN model for detecting brain tumors. CE-MRI benchmark dataset is used for experimental analysis and recorded 94.82% accuracy. Rahman et al. [21] proposed a Smart E-Health care system by employing Fog Computing thus making geo disseminated intermediate intelligence layer among sensors and cloud. Even implemented a smart health gateway called UT GATE and Early Warning Score (EWS) health monitoring system to meet the challenges viz. energy efficiency, security, interoperability, reliability, mobility, and enhanced system intelligence.

The article "A Comprehensive Review on Smart Health Care: Applications, Paradigms, and Challenges with Case Studies" was published in 2022. Journal: Contrast Media Mol Imaging.

Verma et al. [22] proposed an IoT fog cloud-based Cyber-physical system to diagnose and classify ulcerative colitis. For detecting and classifying cancer deep neural networks (DNN) and Naive Bayes classifiers are utilized. The key concept of the proposed system is to generate real-time alarms in emergency conditions (registered patients of the proposed system), and the cloud is employed to store the patient data. Mohamad et al. [23] developed an android system to pronounce and write Hijaiyah letters using a dynamic time-wrapping approach. Voice analogous technique is used for extracting data, inputs, and voice, whereas principal component analysis (PCA) is used for image extraction and MFCC to extract voices. The system recorded 92.85%.

De Brouwer et al. [24] proposed a framework for healthcare systems to communicate data among smart home sensors and smart hospital sensors. The system is used to monitor constantly for clinically diagnosed patients and emergency alarms are responded to accordingly. The key benefit of the system is it eradicates the data latency to enhance the responsiveness of the system. Modu et al. [25] developed a warning system and an android application to analyze malaria outbreaks. For experimental analysis, data are acquired from Climate Forecast System Reanalysis (CFSR). Hypothetical SEM and ellipse shapes are utilized for detecting the ecological factor relationship. SVM, KNN, decision trees, and Naive Bayes machine learning algorithms are utilized for predicting the disease and recorded accuracy between 80.06% and 99.0%. Li et al. [26] developed a system to detect human emotions and a hybrid deep neural network, i.e., CNN and LSTM are employed for this purpose. For experimental analysis, EEG signal data were used. EEG spatial and temporal characteristics were integrated and then converted the outcome into a 2D image. The proposed system recorded 75.2% accuracy.

According to the literature done, Table 2 summarizes deep learning and machine learning techniques incorporated with IoT can be applied for healthcare applications for monitoring, classification, and diagnosis of various diseases like cancer, Alzheimer's, cardiovascular diseases, brain tumor, elderly patient monitoring, and so on. It is observed that the machine learning algorithms performed well for classification purposes and whereas deep learning algorithms worked well for segmentation, detection, and monitoring. SVM, ANN, and CNN have mostly used algorithms, and where they demonstrated that they typically had high evaluation performances.

The article "A Comprehensive Review on Smart Health Care: Applications, Paradigms, and Challenges with Case Studies" was published in 2022. Journal: Contrast Media Mol Imaging.

## 3. Background Study

### 3.1. Machine Learning (ML)

ML is a branch of AI which aims on automating machines with minimum human involvement. It is broadly categorized into three types: supervised learning, unsupervised learning, reinforcement learning, and semi-supervised learning. Supervised and unsupervised algorithms implement mathematical models and are designed to provide proficiency to systems to analyze and learn how to address different tasks. Dataset and corresponding labels (i.e., values, or classes) are used to train the model in supervised learning. Input dataset and its relevant outputs are fed to the algorithm, then it earns through comparing actual output by correct output to identify errors, then accordingly model is modified [41]. Further, it is divided into different methods such as classification, prediction, regression, and gradient boosting. Examples of supervised learning are support vector machine (SVM), linear regression (LR), random forest (RF), and decision trees (DT). Unsupervised learning trains the model only on the given input values; corresponding output variables are not fed to the model along with input data unlike supervised learning, and it is further classified into clustering and association problems which means models are not supervised based on training data, rather it identifies hidden patterns from input data like the human brain. *K*-means, *k*-nearest neighbors (KNN), principal component analysis (PCA), independent component analysis (ICA), hierarchal clustering, and the apriori algorithm are some of the examples of unsupervised algorithms [42]. Whereas semi-supervised learning utilizes both labeled and unlabelled data for training and sometimes, it employs both supervised and unsupervised methods.

ML is advancing promptly in every field due to its advanced algorithms that detect and classify objects. ML in smart healthcare plays a significant role as it advances services provided by healthcare systems such as disease analysis, precise findings, accurate diagnosis, and early-stage prediction. Since medical data are in digital form, to exploit these data in smart healthcare systems, they are numerous challenges to conquer. In recent years, there has been enormous growth in healthcare data which needs to be managed and classified accordingly for accurate diagnosis. ML algorithms can be employed to provide solutions to different healthcare problems.

Research surveys had demonstrated that ML had achieved enhanced performance for disease prediction, diagnosis, and classification tasks. SVM, KNN, RF, and CNN are some of the ML algorithms which fit best for disease classification and identification [43, 44]. Some of the applications of ML in smart healthcare are disease identification, diagnosis, medical image diagnosis, personalized medication, robotic surgeries, cancer detection, oral disease detection, etc.

The article "A Comprehensive Review on Smart Health Care: Applications, Paradigms, and Challenges with Case Studies" was published in 2022. Journal: Contrast Media Mol Imaging.

In [45], the author developed a model (ML based, i.e., ANN and RF) to diagnose and identify bacteria intoxication among serious patients and recorded 90.8% accuracy. In [46, 47], and [48], a system was proposed by utilizing data mining techniques, ensemble learning approach, and SVM respectively to identify readmitting of ICU patients. In [49], a DL model was proposed by employing a CNN algorithm to diagnose glaucoma and obtained 81.6% accuracy on data acquired from Beijing Tongren Hospital. In [50], the authors developed a model by integrating different ML algorithms, i.e., Linear Regression, Lasso Regression, Ridge Regression, and Elastic Net to identify Alzheimer's disease (AD) MMSE scores (Mini-Mental State Examination). A cataract detection model was proposed [51], by employing SVM, and a skating algorithm and obtained around 80% to 84% accuracy. SVM and RF algorithms were utilized for analyzing EHR data [52]. The disease diagnosis model was developed [53] by implementing SVM and deep belief network.

### 3.2. Deep Learning (DL)

DL is a subdomain of ML engrossed by algorithms, functioning like the human brain, i.e., neural networks. The key asset of DL over ML is that it removes the preprocessing, feature extraction, and feature selection processes that are engaged in traditional machine learning. DL algorithms work well for unstructured data such as images, records, text, sensor data, geospatial data, etc., and feature extraction, and feature selection processes are automated. Artificial neural networks or deep neural networks simulate the working of the human brain by employing various elements like inputs, weights, bias, and fusing data, where all these elements function simultaneously to accomplish various tasks in a particular classification, and recognition [54].

Deep learning algorithms consist of three layers input, output, and hidden layer. Input and output layers are known as visible layers, input layers acquire and process the data, whereas the output layer is used to classify or predict the result. The main computations of the network are carried out in the hidden layers. In DL algorithms multiple layers and nodes are interlinked together to optimize and enhance the task of either classification or recognition. Such computation successions over a network are known as “Forward Propagation”. Layers or algorithms where errors are computed through backward traversal by adjusting nodal weights are known as “Backward Propagation”. These two forward and backward propagations enable the algorithm for claiming the predictions accurately.

The article "A Comprehensive Review on Smart Health Care: Applications, Paradigms, and Challenges with Case Studies" was published in 2022. Journal: Contrast Media Mol Imaging.

Since DL algorithms analyze data according to the functioning of the brain, it is feasible to be implemented it in different real-world tasks. It is mostly applied for image, text, and speech recognition, disease detection [55], prediction, and diagnosis, drug discovery, business and management, manufacturing, bioinformatics, and natural language processing. It has been discovered that these applications are unified as a range of services and products such that clients are strangers to the intricate functioning of the model. 

#### 3.2.1. Deep Learning Architectures

Deep learning algorithms give the best performance for all types of data; the key requirements of this algorithm are an enormous amount of data and a high processing unit. Deep learning algorithms are majorly classified into two types of supervised deep learning, i.e., artificial neural networks (ANNs), convolutional neural networks (CNNs), recurrent neural networks (RNNs) and unsupervised deep learning autoencoder, Boltzmann machine and Self Organizing Maps (SOM). These algorithms consist of layers and numerous nodes. Layers can be specified based on the task and different kinds of models had been designed for different tasks like CNNs for recognition tasks, RNNs for time sequence and prediction problems, U-Nets for medical images, and in deep learning it is specified that there is no specific algorithm for a specific task and the algorithm can be structured based on various factors. The following section briefly explains various deep learning algorithms and table 4 describes the summary of various deep learning algorithms and Table 3 describes the summary of various deep learning algorithm.

The term “deep” applies to learning/analyzing succeeding layers from progressive important input images. The depth of the network is determined by the number of layers employed. At present deep learning, architectures include nearly tens to hundreds of layers. The traditional machine learning techniques usually emphasize learning from a few layers, i.e., one or two; these techniques are considered shallow learning.

(i) *Convolutional Neural Networks (CNNs)*. The most prominent deep learning algorithm is CNN, inclusive of several receptive layers enabling robust and fast training to process the input images. It is mainly applied for various computer vision tasks and to enhance the performance of recognition problems [37, 38]. CNNs are neural networks that use both mathematical convolutions and matrices. CNN layers are organized in overlapping forms across the input layers to procure high-resolution outcomes like the original input and every layer in the network follows the above process. The major aim of CNNs is to analyze data-specified kernels in preference to predefined kernels. It employs a sequence of convolutions followed by pooling and activation functions to extract features automatically and activate the neurons, whereas a fully connected layer is employed to classify the extracted features; all CNN operations are depicted in Figure 1.
Inputs of the CNN layer are placed in a three-dimensional matrix, i.e., *hwd* where *h* is the height, *w* is the width, and *d* is the depth of the network.
Several filters of size *m* × *n* (*m* > *d* and *n* ≥ *d*) are present in each layer.
As stated previously, filters are the kernels of network internal connection which are convolved through input and sharing the same parameters, i.e., weight (*W*^*K*^) and bias (*b*^*k*^) to create feature maps *k*(*b*^*k*^) of size *h*^−^*m*^−1^. All the convolutional layers perform the dot product among input and weight. The next activation operation is applied to the convolutional layer outcome, i.e., as follows:
  (1) $$\begin{array}{c} h^{k}=f\left(W^{k}*x+b^{k}\right). \end{array}$$
Next subsampling is done, where all the feature maps are down-sampled for dimensionality reduction thus training is enhanced and regulates overfitting problems, later the pooling function is employed. At last, the fully connected layer acquires the preceding layers' outcome and generates higher-level output, where generally, the softmax function is applied to perform a classification task.
(ii)   *Recurrent Neural Network (RNN).* It is the feed-forward neural network comprising recurrent memory units which acquire and store preceding layer outcomes and feed them to the succeeding layer as input to predict the specific layer output, Figure 2 represents the simple recurrent unit.
In Figure 2, *x* represents the input, *y* represents the output, and *h* is the hidden layer. Parameters of the network are represented by *P*, *Q*, and *R* which enhances the output efficiency. Consider the time “*t*” as an instance then the input is depicted as *x*(*t*) and *x*(*t* − 1).
At any given time, *t*, the current input is a combination of input at *x*(*t*) and *x*(*t* − 1). The output at any given time is fetched back to the network to improve the output. Where *P*, *Q*, and *R* are parameters of the network, *x* is the input and *y* is the output, as shown in Figure 3.
As seen in the figure *x*-input layer acquires and passes the input to the next layer h-middle layer; in this layer several weights, bias, and activation functions can be deployed. RNN will regularize the weights, bias, and activation functions to ensure that all the hidden layers share similar parameters and, therefore, the RNN originates a single hidden layer and employs a loop to it.
(iii) *Autoencoder (AE).*Autoencoders are a specific variant of FFNN holding the same input and output. AEs are trained NNs that replace the data from input to output layers. AE includes three parts viz, encoder, decoder, and code unit. The working rule is according to encoding the input data to a smaller dimension “code”, followed by activation, and then it is decoded out of the representation, i.e., the output is generated. The abstract or compacted input data are known as code or depiction of latent space as depicted in Figure 4. It is a dimensionality reduction algorithm, and the applications are prediction, medical domain, image processing, and drug discovery.
It can be constructed with an encoder, decoder, and loss function operator. Input is passed to the encoder unit a fully connected neural network and generates an encoded code, whereas the decoder is also an artificial neural network that generates the output by decoding the encoded code. The key objective of AE is to generate an output similar to input, i.e., the decoder unit is a reflection of the encoder unit. During this process, AE is optimized and enhanced by diminishing the error rate. Deep AE is generally trained through distinct backpropagation techniques like the conjugate gradient approach. Different variants of autoencoders are also present like; sparse autoencoder, denoising autoencoder, contractive autoencoder, saturating autoencoder, zero-bias autoencoder, and convolutional autoencoder.
(iv) *Generative Adversarial Networks (GANs).* GAN is a semi-supervised or unsupervised model, and they are generative models which generate new data samples like the input. Adversarial GAN term implies that there exists competition among generator and discriminator. It is most broadly implemented in CV and NLP applications. It comprises two NN parts, i.e., the generator and the discriminator presented in Figure 5.
(a) *Generator*: It is an NN, efficient to generate new feasible data instances like original data, and these instances are considered as adverse training instances by the discriminator.
(b) *Discriminator*. This is reliable for classification, i.e., to classify the actual instances from those generated by GANs generator. The discriminator penalizes the generator for generating improbable data.

The generator generates the false instances, and the discriminator promptly learns the generated data and declares it as false data. With the progression of training, it generates an instance that may deceive the discriminator. At last, the discriminator becomes inferior at identifying the actual and the false data and classifies the false data as actual data, thus reducing the network efficiency.

The article "A Comprehensive Review on Smart Health Care: Applications, Paradigms, and Challenges with Case Studies" was published in 2022. Journal: Contrast Media Mol Imaging.

Based on the literature, it is observed that the CNN, variants of CNN, CNN-based algorithms, and combination of CNN with other algorithms had achieved better results when compared to other deep learning and traditional algorithms as shown in Figure 6.

### 3.3. IoT

IoT is a system that comprises devices connected which possess the ability to acquire data and can transfer/exchange data through a wireless network automatically. It permits automated data collection and exchange among a wide variety of industrial sectors. IoT had already been implemented in various fields like industrial automation, agriculture, transportation, construction, supply chain, retail, smart home applications, smart cities, smart grids, and smart parking. Apart from all these fields, it can even be applied to healthcare to perform different tasks ranging from patient data collection to monitoring patients' health [56, 57]. The survey done demonstrates that the existing IoT models work well for data gathering and object controlling/monitoring [32, 58, 59] and, therefore, IoT models can be implemented for health monitoring and reporting the patient condition to appropriate persons like doctors, guardians, medical centers, and to emergency crews [60]. The general IoT architecture comprises different layers such as the data management layer, application layer, middleware layer, network layer, and perception layer.  Figure 7 shows the IoT architecture with different layers and the devices used in each layer.

A survey done during the research demonstrates that patient remote health monitoring (RHM) [61] systems are considerable and the key challenge in these systems is the services that it delivers in various environments. RHM systems are implemented to examine and monitor patients' conditions remotely benefiting patients, hospital staff, and resources [62]. The main aim of such systems is to provide the best healthcare services to rural area patients. Even though this system provides diverse services some challenges that need to be overcome are data privacy and data storage which can be solved by introducing cloud-based IoT healthcare systems. Many researchers had developed such systems as described in the literature study since advancement persists the IoT-based RHM systems growing its popularity and it had become a permanent solution to healthcare systems providing services to rural areas and elderly patients [63]. RHM system can be implemented to provide a diverse variety of services like BP checks, heart rate monitoring, temperature check, diabetes checks, rehabilitation, cancer detection, brain-related diseases, health monitoring, and so on. Therefore, these systems can be developed for different tasks, and they are closely related to the applications of equivalent-enabled technologies.

The article "A Comprehensive Review on Smart Health Care: Applications, Paradigms, and Challenges with Case Studies" was published in 2022. Journal: Contrast Media Mol Imaging.

The major requirements of RHM systems are a variety of sensors and communication devices [64]. Widely used sensors are wearable sensors (wireless or external wearable sensors), vision-based sensors, body sensor networks (BSN), and communication devices are categorized into two types, i.e., short-range communication devices and long-range communication devices [65–71] as described in Tables 4 and 3, demonstrating various sensors used in healthcare applications for acquiring real-time data, and the complete range of all communication devices is also described in Table 5.

### 3.4. Cloud Computing

CC is computing service provision through the Internet ranging from servers to software viz. storage space, networking, data communication service, data security challenges (privacy, security, interoperability, and reliability), data analytics, and software. Cloud can be used in any domain differing from business to healthcare for storing, managing, analyzing, and processing data, and it also provides services to manage real-time software and applications. Cloud service deployment is categorized into three types, i.e., private cloud, public cloud, and hybrid cloud [72]. A private cloud is owned by an individual organization or company, and it is placed at an organization's data center [73]. Private cloud resources can be supplied externally or internally at the organization itself and in this cloud maintenance of infrastructures and services are done on a private network. Public clouds are owned and managed by third-party vendors, for example, Microsoft Azure, Amazon Elastic Compute Cloud (EC2), IBM's Cloud, etc. all the services and resources in the public cloud are maintained by vendors (cloud providers) the user can access these services and resources through Internet browsers [74]. Private and public clouds are integrated to form a hybrid cloud; the hybrid cloud provides the facility to access public cloud services from the private cloud which is known as cloud bursting technology. As shown in Figure 8, cloud renders three service layers viz, Infrastructure as a Service (IaaS), Software as a Service (SaaS), and Platform as a Service (PaaS).

- IaaS (Infrastructure as a Service): according to membership clients are serviced by a virtual environment comprising of virtual, networking, and storage devices. The billing system is also provided to clients where one can demand and pay for the required infrastructure.
- SaaS (Software as a Service): this provides data center and software accessibility based on membership. It manages software installation, update, and recovery; this software can be accessed remotely through the Internet.
- PaaS (Platform as a Service): this provides a platform and interfaces where the clients can create, develop, manage, test, and deploy applications by utilizing the interface provided. It also provides a framework where various users can remotely perform collaborative work.

The article "A Comprehensive Review on Smart Health Care: Applications, Paradigms, and Challenges with Case Studies" was published in 2022. Journal: Contrast Media Mol Imaging.

Since the cloud is abundant in services like data storage, data maintenance, and processing, it can be employed in the healthcare sector for storing patients' data and it is also helpful to provide different remote services to both the patients and hospital staff [75]. CC in healthcare advances the organization's efficiency and simultaneously lowers the cost. It benefits the healthcare system in various terms like ease in medical data storage, sharing, and maintenance, and provides an automatic backend. Since machine learning and deep learning work well and give fine results on large datasets and whenever needed physicians need to access patients' health information; these two challenges of the healthcare system can be met by cloud infrastructure integrated with IoT devices [76]. The two key concerns of a cloud-based IoT system are security, and privacy of data, and it should endorse the deployment of ML and DL models on it.  Figure 9 describes the advantages of the cloud in the healthcare system. Characteristics of cloud-based IoT systems are as follows:

1. Cloud data storage: it is a CC model which stores data on the Internet. To diagnose and analyze any disease, data play a major role; consequently, storing data in a repository (database) are necessary to conduct research. It assists the hospitals and clinics to store a massive number of patient and staff data in a database that can be recovered in case of any disaster. Durability, agility, and anywhere-anytime access to data. Object storage, block storage, and file storage are three types of cloud storage methods. The advantages of cloud storage are information maintenance and management, deployment time, and affordable ownership cost [77].
2. Data processing and analysis: the cloud offers different data processing techniques such as computer offloading, online data processing, electronic data processing, real-time processing, and machine learning; among all these, the most applicable methods are machine learning, specified data mining, and offloading processing. Complex data can be processed by the computational offloading method; it transmits the raw data to the cloud where computational resources are applied for further processing. Data analysis can be performed by employing machine and deep learning techniques such as SVM, KNN, decision trees, random forests, CNN, LSTM, and autoencoders, whereas data mining techniques are utilized for extracting adequate information from repositories. The beneficial impact of deploying high-potential computing integrated with processing on smartphones is the execution of sophisticated algorithms with ease producing accurate and robust outcomes, and the smartphone service life is extended because of fewer internal computations.
3. Data cleaning: noise is a significant modification in image pixel value; while data acquisition and transmission noise are initiated in sensed data which decreases the diagnosis performance, thus there is a need for data cleaning. Filters are used for this purpose; an appropriate filter like a mean filter, median filter, Gaussian filter, and wiener filers can be applied for denoising. Image filtering replaces the pixel value with the average neighbor pixel value and thus filtering smooths out the image.
4. Emergency alert: the sudden downfall of health endangers patients' lives peculiarly in case of dreadful diseases; thus, the emergency warning system is important and becomes a protective safeguard for patients' lives. This challenge can be overcome by the cloud-based IoT system which identifies serious situations by data analysis process and alerts the physicians or guardians eventually.

The article "A Comprehensive Review on Smart Health Care: Applications, Paradigms, and Challenges with Case Studies" was published in 2022. Journal: Contrast Media Mol Imaging.

### 3.5. Fog Computing

Fog computing is a novel approach that extends CC to its networking edge. It is a decentralized computing environment where some devices and services are managed by the smart device at the networking edge and rests are managed at remote data hubs like the cloud. It has been determined that fog computing can be considered a platform/framework to support IoT. Fog is considered an additional layer of a decentralized network and it is intricately connected to CC and IoT. The benefit of adopting fog computing in organizations is that it provides various alternatives for data processing which is the major task in all organizations as shown in Figure 10. For example, in various fields (like hospitals, manufacturing, and business) data should be processed at the initial stage to respond quickly [78]. It is implemented to enhance the system efficiency and to decrease data quantity transferring from physical components to the cloud. Since traditional CC approaches transfer complete data to data centers resulting in latency problems.

Nodes in fog networks are computing, storage devices, and networking devices. The working of fog computing depends on sensors, controllers, and actuators where sensors are utilized to acquire data, controllers transfer data to actuators or any other devices [79]. Then, data are analyzed, optimal patterns are defined by actuators and this information is transmitted to end-users through smartphones. The fog layer in IoT architecture works on data instantly and the delay-sensitive data generated by the user at the edge is analyzed promptly. This instant action minimizes time, and cost, unlike cloud operations. Diverse domain applications can be implemented on fog platforms viz, enterprise, healthcare, transportation, electricity, smart cities, smart buildings, etc. Therefore, fog computing surpasses CC by building up a distributed platform for IoT to address embedded devices and sensors' demands for data storage, analysis, and data processing.

The article "A Comprehensive Review on Smart Health Care: Applications, Paradigms, and Challenges with Case Studies" was published in 2022. Journal: Contrast Media Mol Imaging.

## 4. Smart Healthcare Applications and Challenges

### 4.1. Applications

Smart healthcare applications are software's implemented to generate, gather, maintain, and data related to both patients and health organizations. This data is utilized for performing different tasks like remote patient health monitoring [80], generating patient records, planning treatment, disease detection, sensing patient conditions, and so on. Smart healthcare systems benefit patients, physicians, guardians, healthcare centers, and insurance organizations.

Smart Healthcare System (SHS) is a healthcare service and maintenance system that works with integrated technologies like IoT, wearable devices, Internet for the exchange of information, and it binds the patients, medical staff, healthcare institutions, guardians, and data intelligently into a common platform to assist remotely. It is an aggregate of various areas viz, patient monitoring and management, detection of diseases, prevention, and diagnosis, decision-making systems, virtual assistance, drug discovery, health center management, and assisting drug and medical research. A package of distinct technologies viz, IoT, artificial intelligence, cloud computing, fog computing, edge computing [81, 82], big data, the Internet, sensors, wearable devices, applied sciences, and nanotechnology collectively embodies “smart healthcare”. The SHS will facilitate connection among all concerned bodies and acknowledge that all the associates receive the necessary services. Concisely SHS can be defined as the medical information structure of the top level. Prospects of doctors and patients in healthcare systems are discussed as follows:

- Patients: wearable devices or sensors can be used to control/manage and monitor patient health, remote services, elderly people monitoring, and access to data like records and test reports.
- Doctors: various diagnosis and decision-support systems can be utilized, and can access patient data, and monitor patients.

The article "A Comprehensive Review on Smart Health Care: Applications, Paradigms, and Challenges with Case Studies" was published in 2022. Journal: Contrast Media Mol Imaging.

### 4.2. Challenges

Integration of cloud-based IoT and ML techniques in the medical field set out the signature outcome in everyday life which benefits both the patients and the hospital staff. Despite its benefits for the patients, it also leads to some risky challenges which demand viable solutions. Certain significant challenges are listed as follows [83–87]:

1. Security and privacy: since cloud-based IoT systems are ubiquitous, enhancing fundamental issues like security, privacy and integrity play a key role in the integration of different technologies. To meet various data security challenges like data availability, integrity, and authenticity certain measures should be considered to preserve data stored in the cloud. Personal data theft may occur when these security challenges are not addressed and when data becomes vulnerable to third parties it gets complicated as they can perform unauthorized activities on data. Therefore, a profound security system should be developed for decentralized communication devices among IoT devices and the cloud [88].
2. Quality of services (QoS): this is the foremost paradigm while addressing the overall performance outcome of integrated networks. In the case of enormous data storage and data exchange among IoT devices and cloud/data banks, QoS service maintenance is the paramount challenge. Client demands to cloud platform an effective and robust data management as they might be delay sensitive. Therefore, deploying QoS service in applications prevents data loss. The optimal solution for cloud-based IoT applications is using IPv6 protocol as it provides significant quality features along with QoS assurance.
3. Standard protocol support: as there is no common standard IoT architecture various protocols are used to communicate and transfer data in the network. Despite deploying homogenous nodes' primary protocols like Zigbee, CoAp, 6LOWPAN, and Z-wave remaining heterogeneous, it rises to inconsistent conflicts. This may lead to a major challenge when IoT and cloud are combined. Therefore, there is a need to build standard protocols enabling Cloud-based IoT architectures.
4. Delay and bandwidth-limited: decentralized cloud platforms provide unlimited resources and various services, but it does not assure service access through delay and latency. The solution for an optimum efficiency system is using high bandwidth to transmit data. To eradicate delay and latency issues, a fog computing approach can be implemented as an intermediate layer between IoT and the cloud.

The article "A Comprehensive Review on Smart Health Care: Applications, Paradigms, and Challenges with Case Studies" was published in 2022. Journal: Contrast Media Mol Imaging.

Apart from the above-mentioned challenges, some of them are flexibility and technological advancement, proficiency in the healthcare sector, efficient energy and power consumption, wearable device knowledge, and issues related to hardware during data storing and exchanging such as controlling memory, and system performance.

## 5. Case Studies

### 5.1. Brain Cancer

Uncontrolled division and growth of abnormal cells in any part of the brain is known as Brain cancer. Symptoms and diagnosis of a brain tumor depend on the type of tumor, location, and size. Thus, detecting which part is affected by the tumor is an extremely challenging task in segmenting the cancerous part from the noncancerous part. Several challenges had been addressed by many researchers by using various datasets like BRATS, BTI, and BMI [89, 90]. Some of such works are presented in this section. Guo et al [91] proposed two deep learning algorithms, i.e., 2D-CNN and 3D-CNN for 2D and 3D image datasets. The model was optimized by combing two models' outcomes. Zhao et al. [92] developed a 3D model called as Voxel Classification Model. Fully CNN (FCNN) and Conditional Random Fields (CRF) algorithms were used for training the model and three datasets were used for performance analysis, i.e., BRATS2013, BRATS 2015, and BRATS 2016; the segmentation model was built with T1, T2, T1c, and flair information. Heba et al. [93] proposed a model for classifying brain tumors as per DNN and DWT [94] and PCA was used for feature extraction. Three types of malignant brain tumors were classified, glioblastoma, sarcoma, and metastatic bronchogenic carcinoma; 66 MRI real images were collected from Harvard Medical School website (https://www.med.harvard.edu/AANLIB/home.html). In [95] deep transfer learning models were adopted to build a brain classification model and for feature extraction, GoogleNet was implemented. Three types of brain cancer were classified as meningioma glioma and pituitary tumors. The proposed model addressed the challenge of training the system with higher accuracy using fewer samples. DenseNet201 and deep transfer learning algorithms [96] for multiclass brain tumor classification. Feature selection was done using Entropy–Kurtosis-based High Feature Values (EKbHFV) and Modified Genetic Algorithm (MGA) techniques from BRATS2018 and BRATS2019 datasets [97].

### 5.2. Breast Cancer

A profusion of research has taken place in the last research in the field of breast cancer detection and diagnosis; some of this research are specified in the present section. Spanhol et al. [98] developed a system using CNN variant ALexNet for classifying malignant from benign using histopathological images. In [99] Ertosun and Rubin implemented a model to detect the subsistence of mass in mammography (input) images and later it localizes the mass from those images. A deep learning model was designed in [100] to detect mitosis, feature extraction techniques, i.e., CNN was used, and then the output of this was fed to the SVM classifier to detect the tumor in the breast. A deep contour-aware network was developed for mitosis detection, using breast histopathology scans [101]. Xu et al. [102] proposed a classification model using Stacked Sparse Autoencoder (SSAE) for classifying nuclei from histopathology breast images. A greedy algorithm was used for optimizing the SSAE. Furthermore, breast cancer was detected using a mammography image dataset. In [103, 104] a hybrid model (i.e., CNN + SVM) was developed to detect mass from mammographic scans. CNN was trained using mammogram blemishes and the fully connected layer was used to extract high-level features then these features were used for training the SVM classifier. Kim et al [105] proposed a 3D multi-view using CNN to analyze bilateral features using Digital Breast Tomosynthesis (DBT). Volume of Interest (VOI) was obtained from the input volume and to extract features from VOI two different CNN algorithms were implemented. Yu et al. [106] proposed a deep learning-enabled breast cancer diagnosis system for remote healthcare via the 5 G mechanism. The proposed technique is carried out in three steps: first the input is acquired from hospitals through 5 G technology, then a transfer learning algorithm is applied to procure a diagnostic system. At last, this model is deployed on an edge server for remote diagnosis.

The article "A Comprehensive Review on Smart Health Care: Applications, Paradigms, and Challenges with Case Studies" was published in 2022. Journal: Contrast Media Mol Imaging.

### 5.3. Diabetics Detection

Diabetes is an incurable and long-lasting illness caused due to increase in glucose in the blood and it has become increasingly common among people irrespective of sexual orientation, race, age, habits, etc. The primary energy means is glucose and the pancreas secreted hormone, i.e., insulin regulates the metabolism of the body and controls the glucose level in the blood. The body converts the sugar into energy with the help of insulin and stores the excess. If ample insulin is not produced in the body diabetes is caused as blood glucose cannot be regulated and remains in the blood. If the blood glucose level exceeds a minimal value, it leads to various diseases. According to medical research, diabetes is not completely curable, but it is treatable and if it is left untreated it emerges into various diseases viz., heart stroke, brain stroke, kidney failure, blindness, and even may lead to death. Thus, it is requisite to detect diabetes at its early stage, thereby diagnosing and treating it to prevent disease advancement as it aids to death and further diseases. Immense research is going on detecting and diagnosing diabetes at its early stage. Vast medical data can be found through various resources like lab reports, medical images, Electronic Health Record (EHR), and clinical reports but the significant challenge is data understanding and interception. Several methods and techniques are proposed for diabetic detection. In [107] different machine learning techniques had been applied viz, SVM, decision tree, and Naive Bayes, and in [108] a hybrid method is used, i.e., Principal Component Analysis and Adaptive Neuro-Fuzzy Interface System (PCA and ANFIS). ResNet is developed in [109] to address the vanishing gradient problem. ANN architecture is proposed to predict diabetics in [110]; the proposed model is used to minimize the error rate of the function during training and recorded 87% accuracy in prediction, and the estimated error rate is 0.01%. In [111], a computer-aided system had been developed to detect diabetic retinopathy by using digital signals from retinal images. The major aim of the work is to classify nonproliferative diabetic retinopathy from retinal images. [112] CNN approach is developed for segmenting blood vessels of diabetic patients followed by the classification, and then extraction of discriminant patterns is done. [113] A shallow CNN framework is developed. In [114], residual network is developed to classify the retinopathy images automatically.

The article "A Comprehensive Review on Smart Health Care: Applications, Paradigms, and Challenges with Case Studies" was published in 2022. Journal: Contrast Media Mol Imaging.

## 6. Conclusion

Advancement and increasing superiority of cloud-based IoT and DL techniques had become the key elements of healthcare applications. Cloud and IoT integration in the healthcare sector is mostly recommended due to its effective services like immense data repositories, data availability, optimum performance, network balancing, and computing infrastructures. Most of the research had been done on cloud-based IoT healthcare systems emphasizing background technologies, and system architectures. This study presents an intense review of cloud and IoT integration with machine learning and deep learning techniques in healthcare. We reviewed the literature thoroughly and preferred significant and contemporary studies to determine the techniques and research gaps. This study also presents cloud services, and advantages in healthcare, IoT architecture, various communication protocols, sensors, ML, and DL techniques, and challenges. In addition, a thorough analysis of their advantages and disadvantages, and challenges are discussed. This study gives an insight to the researchers and can exert them the opportunity to begin their research by choosing an application/domain from the available methods discussed. With adequate adherence to security and privacy measures, the cloud-based IoT and ML healthcare systems are accurate and of complete assistance to patients, guardians, and hospital staff.

The article "A Comprehensive Review on Smart Health Care: Applications, Paradigms, and Challenges with Case Studies" was published in 2022. Journal: Contrast Media Mol Imaging.

## Figures and Tables

**Figure 1:** Architecture of CNN, representing all the operations of CNN, i.e., convolution, pooling, feature extraction, and classification with “*n*” number of convolution, pooling, and fully connected layers.

**Figure 2:** Simple recurrent unit representation of RNN.

**Figure 3:** The architecture of a recurrent neural network, where *P*, *Q*, and *R* are parameters of the network, *x* is the input and *y* is the output.

**Figure 4:** Autoencoder architecture.

**Figure 5:** Generative adversarial networks (GAN).

**Figure 6:** Comparison of deep learning algorithms, i.e., CNN, RNN, AE, and GAN performance.

**Figure 7:** IoT layered architecture.

**Figure 8:** Cloud services—IaaS, PaaS, and SaaS.

**Figure 9:** Advantageous of cloud in healthcare.

**Figure 10:** Fog computing architecture.

**Table 1:** list of abbreviations.

Abbreviation	Definition
6LoPWAN	IPv6 over low-power wireless personal area networks
AD	Alzheimer's disease
AE	Autoencoder
AID	Automated insulin delivery
ANN	Artificial neural network
BMI	Body mass index
BSN	Body sensor network
CAE	Convolutional autoencoder
CART	Classification and regression trees
CC	Cloud computing
CE-MRI	Contrast-enhanced magnetic resonance imaging
CFSR	Climate forecast system reanalysis
CNN	Convolutional neural network
CoAP	Constrained application protocol
CRF	Conditional random fields
CV	Computer vision
DBN	Deep belief network
DL	Deep learning
DNN	Deep neural network
DT	Decision tree
DTW	Dynamic time warping
DWT	Discrete wavelet transform
EC2	Amazon elastic compute cloud
EEG	Electroencephalogram
EHR	Electronic health record
EKbHFV	Kurtosis-based high feature values
EMR	Electronic medical record
EWS	Early warning system
FFNN	Feed forward neural network
GAN	Generative adversarial network
GFB	Grey filter Bayesian
HAR	Human action recognition
IaaS	Internet as a service
IBM	International business machines
IoT	Internet of things
ICA	Independent component analysis
*K*-NN	*K*-nearest neighbor
LAD	Logical analysis of data
LR	Logistic regression
LSTM	Long short-term memory
MGA	Modified genetic algorithm
MHEALTH	Mobile-health
ML	Machine learning
MMSE	Mini-mental state examination
MRI	Magnetic resonance imaging
NLP	Natural language processing
PaaS	Platform as a service
PCA	Principal component analysis
QoS	Quality of service
REP	Reduced error pruning
REST	Representational state transfer
RF	Random forest
RFID	Radio-frequency identification
RHM	Remote healthcare monitoring
RNN	Recurrent neural network
SaaS	Software as a service
SHMS	Smart healthcare monitoring system
SHS	Smart healthcare system
SOM	Self-organizing maps
SVM	Support vector machine
UHF	Ultra-high frequency
VOI	Volume of interest
WiFi	Wireless fidelity
WSN	Wireless sensor network

The article "A Comprehensive Review on Smart Health Care: Applications, Paradigms, and Challenges with Case Studies" was published in 2022. Journal: Contrast Media Mol Imaging.

**Table 2:** Summary of deep learning-based algorithms applied for various disease detection and classification.

Reference	Algorithms used	Application	Accuracy
[27]	CNN	Alzheimer disease diagnosis	97%
[28]	CNN	COVID-19 detection	99%
[29]	DNN	To detect COVID-19	99.7%
[30]	DBM	Cancer diagnosis	95.5%
[31]	DBN	Classification of COVID-19	90%
[32]	ANN + CNN + LSTM	Walking behavior detection	96%
[33]	CNN + CAE + DAE	Fall detection	99.9%
[34]	Faster RCNN	Remote healthcare system	Faster RCNN outperformed fast RCNN and RCNN
[35]	Deep ensemble learning	Cardiovascular disease detection	98.62%
[36]	MobileNet	Skin cancer detection	91.25%
[37]	Deep CNN	Skin carcinoma classification	93.16%
[38]	Capsule network	Brain tumor classification	86.56%
[39]	Pretrained CNN models	Breast cancer detection and classification	98.96%
[40]	CNN + DarkNet-53	Breast cancer classification	99.1%

**Table 3:** Summary of various deep learning algorithms and their advantages and disadvantages.

DL algorithm	Description	Advantages	Disadvantages	Applications
MLP	MLP is a feed-forward neural network that maps input set to relevant output. It is a confined acyclic graph where nodes are neurons with logistic activation functions.	can solve complex nonlinear problems with limited data, i.e., fewer parameters.	The outcome of the model depends on the model training. More processing time.	Classification, recognition, business, self-driving, prediction, etc.

CNN	CNN is a variant of ANN which is mostly used for image processing and recognition tasks peculiarly destined for processing pixel data.	Relevant information is only retrieved. Outperforms accurate accuracy for image processing.	Enormous data for training and more computational cost.	Image, speech and pattern recognition and processing, video analysis, and natural language processing

RNN	It's an expansion of the feed-forward neural network. A variant of ANN includes loops and memory units that store information, and it utilizes sequential and time-series data.	Remembers the information, weights are used throughout the timestamp and can be implemented along with CNN to prolong the neighborhood pixel efficiency.	Vanishing gradient problem, difficulty in training, slow computation, complex while training parallel process	Temporal problems, prediction, machine translation, video captioning, speech recognition, robot control, and so on

LSTM	LSTM is a type of RNN appropriate to learn order dependency in time sequence prediction problems. Like RNN information can be stored.	Supervise the vanishing gradient problem, a substantial range of parameters, and no limit to input length.	Slow computation, difficulty while accessing previous information, not interpretable	Sequence prediction problems, sentiment analysis, grammar learning, semantic parsing, speech recognition, and so on

DBN	A variant of generative neural network. DBN is trained by employing a greedy algorithm and it utilizes the layer-by-layer approach to learn top-down models.	Capable of using hidden layers efficiently. Capable of learning features acquired from layered learning approaches. Work well for unlabelled data, robustness in classification.	High runtime complexities are not an appropriate outcome while working with pretrained algorithms	Image classification, audio classification, speech recognition, natural language processing language translation, expert systems, decision support system

AE	Is a neural network that employs the backpropagation technique for feature learning. It consists of two blocks, i.e., encoding and decoding.	Works well for compression and dimensionality reduction problems, features learned by one autoencoder network can be applied to another problem.	Inefficient for image reconstruction. For complex images outcome results in a blurry image.	Clustering, image coloring, feature variation, dimensionality reduction, denoising images, watermark removal

GAN	Is a DNN architecture that is capable of learning from the training dataset and generates new datasets like the original data.	Generates similar outcome to original data, easy data interpretation, and an efficient algorithm for the recognition task	Difficult to train, the learning process contains missing patterns thus model may collapse	Data and image generation, image conversion, automatic model generation, text to image translation, semantic image to photo translation

The article "A Comprehensive Review on Smart Health Care: Applications, Paradigms, and Challenges with Case Studies" was published in 2022. Journal: Contrast Media Mol Imaging.

**Table 4:** Various sensors are utilized in healthcare to sense and acquire data.

Sensors	Biosignal type	Function
Temperature	Body temperature	Body or device temperature is measured
Accelerometer	Body movement	Acceleration force is measured
Gyroscope	Angle rotation, vibration, and axis	The rotation rate of the device is measured
Pulse oximeter	Oxygen saturation	Measures level of oxygen in the blood
Magnetic sensors	Body motion, and position parameters	Measures surroundings magnetic field
Chest electrodes	ECG	Heartbeat measurement
Phonocardiograph	Cardiac auscultation	Cardiac auscultation measurement by using a stethoscope
Piezoelectric sensor	Breathing rate	Measures breathing rate
Electrodes	Electrodermal activity	Measures cardiac health condition
Optical infrared thermopile	Photo-plethysmography, and skin temperature	Measures quality of sleep, and stress
Global positioning sensors	Physical activities	Measures human physical activity
Force sensors	Kidney dialysis	Employed in kidney dialyzing devices
Implantable pacemaker	Heart rhythm	Provides synced electric stimulus heart rhythm to the heart muscle to figure control heart rhythm
Pressure sensor	Sleep disorders, BP control	Monitors BP, employed in sleep apnea devices and infusion pumps
Glucometer	Glucose concentration	Measures glucose concentration in blood
Electroencephalogram sensor	EEG	Measures brain electrical activity
Electromyogram sensor	Skeletal muscles	Measures electrical activity of skeletal muscles
Airflow sensors	Heart pumps, laparoscopy, etc.	Employed in various devices like heat pumps, anesthesia delivery devices, laparoscopy, etc.

**Table 5:** Short- and long-range communication devices.

Communication devices		Range	Topology	Band of operation	Data rate	Security	Employability in HCS
Short-range communication devices	Bluetooth zigbee 6LoWPAN	150 m 30 m 10–100 m	Star mesh mesh	2.4 GHz 2.4 GHz 868 & 915 MHz, 2.4 GHz	1 Mbps 250 kbps 250 kbps	128-AES encryption Optional128-AES encryption end-to-end hop-by-hop	High moderate moderate

	*Z*-wave	100 m	Mesh	908.4 HGz	100 kbps	128 Bit zero temporary key	Moderate

Long-range communication devices	SigFox LoRa NB-IoT	9.5 km 7.2 km 15 km	Hop-star star-of-stars mesh to star	868 MHz 868 MHz LTE	100 bps 0.25–5.5 kbps 250 kbps	Private key unique key 3 GPP S3 security	Low moderate high

## Data Availability

Data set will be provided upon request.
